The article "Deep Learning-Based Ultrasound Combined with Gastroscope for the Diagnosis and Nursing of Upper Gastrointestinal Submucous Lesions" was published in 2022. Journal: Comput Math Methods Med.

# Deep Learning-Based Ultrasound Combined with Gastroscope for the Diagnosis and Nursing of Upper Gastrointestinal Submucous Lesions

**DOI:** 10.1155/2022/1607099

**Published:** 2022-04-19

**Authors:** Lima Xia, Suhua Sun, Weijie Dai

**Affiliations:** Department of Endoscope Center, The Affiliated Huaian No.1 People's Hospital, Nanjing Medical University, Huaian, 223300 Jiangsu, China

## Abstract

The study focused on the diagnostic value of deep learning-based ultrasound combined with gastroscope examination for upper gastrointestinal submucous lesions and nursing. A total of 104 patients with upper gastrointestinal submucous lesions diagnosed in hospital were selected as the research subjects. In this study, the feed forward denoising convulsive neural network (DnCNN) was improved, and the n-DnCNN model was designed and applied to ultrasonic image processing. The peak signal-to-noise ratio (PSNR) and structural similarity (SSIM) of Gaussian filtering, NL-means, and DnCNN were then compared with n-DnCNN. Subsequently, the distribution and types of submucosal lesions in different parts of the upper digestive tract were analyzed by ultrasound combined with gastroscope and gastroscope examination alone, and the diagnostic performance of this method was evaluated. The results showed that the average PSNR and SSIM of the n-DnCNN model were 33.01 dB and 0.87, respectively, which were significantly higher than GF, NL-means, and DnCNN algorithms, and the difference was statistically significant (*P* < 0.05). Of the 116 lesions detected, 49 were located in the esophagus (42.24%), 52 in the stomach (44.83%), and 15 in the duodenum (12.93%). Of the 49 esophageal submucosal lesions, 6.12% were located in the upper esophagus, 55.1% in the middle esophagus, and 38.79% in the lower esophagus, and the difference was statistically significant (*P* < 0.05). Of the gastric submucosal lesions, the lesions in the gastric cardia were significantly less than in other parts, and the difference was statistically significant (*P* < 0.05). The accuracy of ultrasound combined with gastroscope in the diagnosis of upper gastrointestinal submucous episodes was 82.32%, higher than that of gastroscope examination, and the difference was statistically significant (*P* < 0.05). In conclusion, the n-DnCNN model has a good noise reduction effect, and the obtained image is of high quality. Ultrasound combined with gastroscope examination can effectively improve the accuracy of diagnosis of upper gastrointestinal submucous lesions.

## 1. Introduction

Upper gastrointestinal submucous lesions usually refer to the protrusion lesions covered by a normal mucous membrane in the upper gastrointestinal tract, manifesting as smooth and continuous spherical or semispherical swelling under a gastroscope, mainly including stromal tumor, leiomyoma, cyst, lipoma, and hemangioma [1, 2]. The lesion lacks specificity. A tissue biopsy can only be performed on the mucosa and cannot determine the nature of the lesion. Conventional imaging examinations such as computed tomography (CT) and magnetic resonance imaging (MRI) have low sensitivity, specificity, and accuracy, which cannot meet the requirements for clinical treatment and prognosis evaluation of upper gastrointestinal submucous lesions [3, 4].

With the development of imaging technology, Endoscopic Ultrasound (EUS) has become the primary method for diagnosis and evaluation of upper gastrointestinal submucous lesions [5, 6]. This is a new technology that combines a gastroscope with ultrasound. Specifically, the miniature high-frequency ultrasound probe is placed at the top of the gastroscope. When the gastroscope enters the human body, the conditions in the digestive tract, including the changes in tissue, surface morphology, and blood vessels, can be directly observed through the gastroscope, and the ultrasonic probe at the top of the gastroscope can also be used to scan and obtain the surrounding tissue and blood vessel structure images of the scanned part [7–9]. This method is easy to operate, can clearly show the hierarchical structure of the inner wall of the digestive tract, and can reflect the accurate location of lesions [10]. Additionally, this method can also biopsy the lesion site by guided fine needle aspiration, which provides reliable imaging and pathological data for the clinical diagnosis and treatment of upper gastrointestinal intentional submucous lesions [11–14].

With the rapid development of imaging technology, high-quality medical images have become an important reference for the clinical diagnosis and treatment of diseases [15]. However, there are noise and false texture in conventional ultrasound images, which cause visual interference and seriously affect doctors' judgment [16]. Some scholars use the nonlocal total variation (NLTV) method to effectively remove the acoustic speckle. Deep learning technology has been well developed and applied in image processing, which effectively improves the accuracy of image recognition and the detection of target edges [17, 18].

To sum up, considering the lack of specificity of upper gastrointestinal submucous lesions in imaging and the improvement and development of deep learning technology in imaging, the deep learning technology was adopted in the diagnosis and evaluation of upper gastrointestinal submucous lesions by ultrasound combined with gastroscope and compared with Gaussian filtering, NL-means, and DnCNN models, so as to comprehensively evaluate the clinical diagnostic value of this method in upper gastrointestinal submucosal lesions and nursing care and provide effective data support for clinical diagnosis.

## 2. Materials and Methods

### 2.1. Research Subjects

A total of 104 patients with upper gastrointestinal submucous lesions diagnosed in hospital from May 2018 to June 2020 were selected as the research subjects, including 51 males and 53 females, aged from 23 to 82 years, with an average of 46.32 ± 12.3 years. General clinical data of the patients were collected, and all patients underwent general gastroscope and ultrasound combined gastroscope examination. This study had been approved by the ethics committee of the hospital. Patients and their families had known about this study and signed the informed consent form.

Inclusion criteria include (1) patients who met the diagnostic criteria of submucosal lesions of the upper digestive tract, (2) age over 18 years, and (3) no contraindications of ultrasound and gastroscopy.

Exclusion criteria include (1) combination with serious cardiopulmonary diseases, (2) with contraindications for ultrasound and gastroscope examination, (3) patients with thoracic and abdominal aortic aneurysms, and (4) those with serious mental disorders who cannot cooperate in the experiment.

### 2.2. Imaging Examination

The color Doppler ultrasound diagnostic instrument with a probe frequency of 2-12 mHz was used for ultrasonic examination. During the examination, the patient was in a supine position. The ultrasonic probe was placed in the upper digestive tract. The high-frequency probe, together with the local amplification function, was used to observe the size, position, shape, surrounding tissue, echo intensity, echo internal homogeneity, and boundary. For gastroscope examination, the lens entered into the upper digestive tract for a comprehensive and careful examination to observe and record the lesion location, size, and shape.

### 2.3. Nursing Methods

*Preoperative nursing*: nurses collected the general clinical data of patients before surgery to identify the lesion site and nature of upper gastrointestinal submucous lesions. Then, blood routine and liver and kidney function examinations were performed, and the blood type was identified for blood preparation. Psychological nursing was carried out to relieve tension, anxiety, and fear of patients. An infusion valve was then constructed for fluid infusion.

*Intraoperative cooperation*: in a decubital supine position, the patient was observed for vital signs and actively cooperated with surgeons to complete the surgery.

*Postoperative care*: low-flow oxygen inhalation and continuous ECG monitoring were given in accordance with the doctor's advice, and patients' vital signs and wound conditions were observed. The patient stayed in bed on the first day after surgery and avoided forced movements such as defecation, coughing, and expectoration. Antibiotics, hemostatic drugs, and proton pump inhibitor were given in accordance with the doctor's advice. According to the specific situation of the patient, the patient was instructed to fast for 1 day after the operation and eat a liquid diet for 3 days. During the transition from a liquid diet to a normal diet, the patients should eat 5-6 smaller meals and avoid eating rough and hard food.

### 2.4. Improvement of DnCNN

The ultrasound imaging is based on the divergence, diffraction, and refraction of ultrasound when it encounters different tissue. The noise of ultrasound imaging mainly arises from the interference of ultrasound. If *D*_1_ and *D*_2_ are the whole amplitude of two different acoustic waves and *l* is the difference of wave paths, the combined amplitude of the two acoustic waves can be expressed as follows:

(1) $$\begin{array}{c} D=\sqrt{D_{1}^{2}+D_{2}^{2}+2D_{1}D_{2}\cos\frac{2\pi l}{D}}. \end{array}$$

Under ideal conditions, speckle noise distribution conforms to Rayleigh distribution, which can be expressed as follows:

(2) $$\begin{array}{c} g\left(m\right)=\frac{z}{\sigma^{2}}\exp\left(-\frac{z^{2}}{2\sigma^{2}}\right). \end{array}$$

Considering the complexity of speckle noise in ultrasound imaging, Equation (3) is constructed to represent noise:

(3) $$\begin{array}{c} g\left(m,n\right)=k\left(m,n\right)*p_{1}\left(m,n\right)+p_{2}\left(m,n\right), \end{array}$$

where *g*(*m*, *n*) denotes sonogram containing noise, *k*(*m*, *n*) represents the label image without noise, *p*_1_(*m*, *n*) represents multiplicative noise, and *p*_2_(*m*, *n*) represents additive noise.

Based on DnCNN, the n-DnCNN model is designed in this study. The improved algorithm structure is shown in Figure 1. In this study, ReLu function is introduced in the first and 15th convolutional layers and BN function and ReLu function are used in the 2nd to 15th convolutional layers to extract noise information. Finally, the activated function Tanh outputs the denoised image. The improved algorithm overcomes the problem of difficult convergence in the training of CNN.

### 2.5. Observation Indicators

In the study, peak signal-to-noise ratio (PSNR) and Structural Similarity Index Measurement (SSIM) are introduced to evaluate the quality of the image. Gaussian filtering (GF) [19], nonlocal means (NL-means) [20], and DnCNN [21] are compared for PSNR and SSIM.

PSNR represents the amount of noise in the image after denoising. A higher PSNR value indicates less noise in the image and better denoising effects. Its equation is derived from the Root Mean Square Error (RMSE) equation:

(4) $$\begin{array}{c} \text{RMSE}=\frac{1}{x\times y}\underset{q=1}{\overset{x}{\Sigma }}\underset{r=1}{\overset{y}{\Sigma }}{\left(\overset{\wedge }{s}\left(q,r\right)-s\left(q,r\right)\right)}^{2}, \end{array}$$

(5) $$\begin{array}{c} \text{PSNR}=10\log_{10}\frac{{\left(2^{n}-1\right)}^{2}}{\text{RMSE}}, \end{array}$$

where *A*(*q*, *r*) is the target image, *B*(*q*, *r*) is the original image, *X* represents pixels on the horizontal axis of the image, and *Y* represents pixels on the vertical axis. SSIM is mainly used to compare the similarity between two images to judge the similarity of image content. A larger SSIM value indicates higher similarity and quality of images. It is expressed as follows:

(6) $$\begin{array}{c} \text{SSIM}\left(P,Q\right)=\frac{\left(2\alpha_{P}\alpha_{Q}+G_{1}\right)\left(2\rho_{PQ}+G_{2}\right)}{\left(\alpha_{P}^{2}+\alpha_{Q}^{2}+G_{1}\right)\left(\rho_{P}^{2}+\rho_{Q}^{2}+G_{2}\right)}, \end{array}$$

where *P* denotes the original image, *Q* denotes the images to be compared with, (*α*_*P*_, *α*_*Q*_) is the brightness of the image, (*ρ*_*P*_, *ρ*_*Q*_) is the contrast of the image, and *ρ*_*QP*_ denotes the structure of the image.

### 2.6. Statistical Methods

SPSS2.0 software is adopted for the statistical analysis of the experimental data. The experimental data is expressed as the mean ± standard deviation (*x* ± *s*). The measurement data is according to normal distribution, and the *f* test uses the *t* test for comparison between two samples. The classification of data employs the *χ*^2^ test, and *I*^2^ is used to assess the size of the heterogeneity. *P* < 0.05 indicates a statistically significant difference.

## 3. Results

### 3.1. Analysis of the Algorithm Performance

During the training of the algorithm, the multiplicative Gamma noise was added to the images of the training set. A total of 48 images with Gamma noise were trained in the study. The average PSNR and SSIM before and after denoising were compared, as shown in Figure 2. It was noted that the average PSNR and SSIM of the image after denoising were significantly higher than those before denoising, and the differences were statistically significant (*P* < 0.05). It indicated that the n-DnCNN model designed in this study had a good denoising effect on multiplicative noise.

After verifying the denoising effect of the improved algorithm, the study compared the denoising effect of Gaussian filtering, NL-means, and DnCNN of 300 test images. As shown in Figure 3, the average PSNR and SSIM of the n-DnCNN model were 33.01 dB and 0.87, respectively, significantly higher than other algorithms, and the difference was statistically significant.

Figure 4 shows the denoising effects of the four algorithms on the ultrasound images of gastric leiomyoma and gastric stromal tumors. It was noted that the denoising effect of the n-DnCNN model was significantly better than that of filtering, NL-means, and DnCNN and that the images obtained were the clearest, with good PSNR and SSIM values.

### 3.2. Distribution of Upper Gastrointestinal Submucous Lesions

A total of 104 patients were included in the study, including 51 males and 53 females. A total of 116 upper gastrointestinal submucous lesions were detected, and Figure 5 shows their distribution in the upper gastrointestinal tract. Of them, 49 (42.24%) were located in the esophagus, 52 (44.83%) in the stomach, and 15 (12.93%) in the duodenum.

Of the 49 lesions in the esophagus, 3 (6.12%) were located at the upper esophagus, 27 (55.1%) at the middle esophagus, and 19 (38.79%) at the lower esophagus. As shown in Figure 6, those located in the upper esophagus were significantly less than those located in the terminal and lower segments, and the difference was statistically significant (*P* < 0.05), while those located in the middle esophagus were the most common.

Of the 52 upper gastrointestinal submucous lesions in the stomach, 5 (9.61%) were located at the gastric cardia, 18 (34.62%) were located at the bottom of the stomach, 14 cases (26.92%) were located in the gastric body, and 15 cases (28.85%) were located in the gastric antrum. As shown in Figure 7, the lesions in the gastric cardia were significantly less than those in other parts, and the difference was statistically significant (*P* < 0.05). The lesions in the gastric fundus were the most, followed by gastric antrum and gastric body.

Of the 15 upper gastrointestinal submucous lesions of the duodenum, 7 (46.67%) were located at the bulb and 8 (53.33%) at the lower duodenum, showing no statistically significant difference (*P* < 0.05) (Figure 8).

### 3.3. The Site and Type of Upper Gastrointestinal Submucous Lesions

A total of 116 lesions were counted in the study, and Figure 9 shows the sites and types of submucosal lesions in the esophagus, stomach, and duodenum.  Figure 9(a) shows 3 leiomyomas on the upper esophagus, 24 leiomyomas and 3 cysts on the middle esophagus, and 18 leiomyomas and 3 cysts on the lower esophagus. It was noted that leiomyomas were more common than the cysts in the esophagus and that leiomyomas located in the upper esophagus were less than those in the middle and lower segments, and the differences were statistically significant (*P* < 0.05).  Figure 9(b) shows 1 leiomyoma and 4 stromal tumors located at the cardia; 1 leiomyoma, 4 stromal tumors, 2 lipomas, 1 ectopic pancreas, and 1 cyst in the gastric fundus; 1 leiomyoma, 11 stromal tumors, and 2 ectopic pancreases in the gastric body; and 1 stromal tumor, 2 lipomas, and 13 ectopic pancreases in the gastric antrum. It was noted that stromal tumors in the fundus and body of the stomach were significantly more than those in other parts and that ectopic pancreas in gastric antrum was significantly more than in other parts, with statistical significance (*P* < 0.05).  Figure 9(c) shows 2 stromal tumors, 4 lipomas, 1 ectopic pancreas, 7 cysts, and 1 adenoma in the duodenum.

### 3.4. Ultrasound Combined with Gastroscope for the Diagnosis of Upper Gastrointestinal Submucous Lesions

In this study, the pathological diagnosis was used as the standard to compare the diagnostic effects of ultrasound combined with gastroscope and gastroscope alone on upper gastrointestinal submucous lesions. As shown in Figure 10, the accuracy of ultrasound combined with gastroscope in the diagnosis of leiomyoma, stromal tumor, lipoma, ectopic pancreas, and cyst was higher than that of gastroscope. The overall accuracy of ultrasound combined with gastroscope for the diagnosis of upper gastrointestinal submucous lesions was 82.32%, which was significantly higher than that of gastroscope, and the difference was statistically significant (*P* < 0.05).

## 4. Discussion

The clinical symptoms of upper gastrointestinal submucous lesions are not specific, and the incidence increases year by year with the changes in living habits and dietary structure [22]. The lesions are divided into benign, malignant potential, and malignant ones, while leiomyoma, stromal tumor, lipoma, ectopic pancreas, and cyst are more common [23]. Because the lesion site is often covered by normal mucosa, it is difficult for a routine biopsy to achieve an accurate diagnosis. The development of ultrasound technology has brought benefits to the clinical diagnosis of upper gastrointestinal submucous lesions, especially EUS technology, which combines ultrasound examination with gastroscope examination and can clearly observe the size, boundary, echo characteristics, and origin of digestive tract lesions [24, 25]. Akahoshi et al. [26] found that the safety and accuracy of EUS were higher than that of ordinary gastroscope examination. In this study, an ultrasound combined with gastroscope model based on deep learning was proposed to evaluate the diagnostic value for upper gastrointestinal submucous lesions and nursing. The n-DnCNN model was designed based on DnCNN and compared with Gaussian filter, NL-means, and DnCNN. The results showed that the average PSNR and SSIM of the n-DnCNN model were 33.01 dB and 0.87, respectively, which were significantly higher than the other three algorithms, and the difference was statistically significant (*P* < 0.05), which showed that the n-DnCNN model had better denoising effect. The research of Jiang et al. [27] showed that the training model of DCNN is generally applicable and has obvious denoising effects, which was in line with the results of this study.

The study is aimed at exploring the diagnostic performance of ultrasound combined with gastroscope examination based on the n-DnCNN model for upper gastrointestinal submucous lesions. First, 104 patients were included, and 116 upper gastrointestinal submucous lesions were detected. Of them, 49 lesions are located in the esophagus (42.24%), 52 lesions are located in the stomach (44.83%), and 15 lesions are located in the duodenum (12.93%). Of the 49 lesions in the esophagus, 3 leiomyomas are on the upper esophagus, 24 leiomyomas and 3 cysts are on the middle esophagus, and 18 leiomyomas and 3 cysts are on the lower esophagus. It was noted that the lesions in the upper esophagus were significantly less than in the terminal and lower esophagus, and the difference was statistically significant (*P* < 0.05). The lesions in the gastric cardia were significantly less than in other parts, and the difference was statistically significant (*P* < 0.05). The lesions in the gastric fundus were the most, followed by the gastric antrum, and finally the gastric body. Of the duodenal submucosal lesions, 7 were located in the bulbar part (46.67%) and 8 in the descending part of the duodenum (53.33%), and there was no significant difference between them (*P* < 0.05). On this basis, the study further explored the distribution and pathological classification of submucosal lesions in various parts. The results showed that leiomyomas in the esophagus were significantly more than cysts, and leiomyomas in the upper esophagus were significantly less than those in the middle and lower esophagus, and the difference was statistically significant (*P* < 0.05). There were more stromal tumors in the bottom and body of the stomach than in other parts, and the ectopic pancreas in the antrum was significantly more than that in other parts, and the difference was statistically significant (*P* < 0.05), which was consistent with the result of Khoury et al. [28]. At last, the study compared the diagnostic effects of ultrasound combined with gastroscope on upper gastrointestinal submucous occasions. The results showed that the accuracy of ultrasound combined with gastroscope in diagnosing upper gastrointestinal submucous lesions was 82.32%, significantly higher than that of gastroscope examination alone, and the difference was statistically significant (*P* < 0.05).

## 5. Conclusion

The study was intended to explore the diagnostic value of ultrasound combined with gastroscope examination based on deep learning for upper gastrointestinal submucous lesions and nursing. The n-DnCNN model was designed based on DnCNN and then compared with Gaussian filter, NL-means, and DnCNN for noise reduction effect. Next, the diagnostic performance of ultrasound combined with gastroscope examination was compared with that of gastroscope examination alone. The results showed that the n-DnCNN model has a good noise reduction effect, and the obtained images are of high quality. Ultrasound combined with gastroscope examination can effectively improve the accuracy of diagnosis of upper gastrointestinal submucous lesions. However, some limitations in the study should be noted. The sample size is small, which will reduce the power of the study. In the follow-up, expanded sample size is necessary to strengthen the findings of the study. In conclusion, this study provides a theoretical basis for the application of deep learning in the field of imaging and the clinical diagnosis of upper gastrointestinal submucosal diseases.

## Figures and Tables

**Figure 1:** The structure of the improved algorithm.

**Figure 2:** Gamma noise experiments. ∗ represents statistically significant difference compared with that before denoising (*P* < 0.05).

**Figure 3:** Comparison of algorithm performance on the test set. ∗ represents a statistically significant difference compared with other algorithms (*P* < 0.05).

**Figure 4:** Denoising effects of different algorithms.

**Figure 5:** Distribution of upper gastrointestinal submucous lesions.

**Figure 6:** Distribution of esophageal submucosal lesions. ∗ represents a statistically significant difference compared with esophageal mucosal lesion distribution (*P* < 0.05).

**Figure 7:** Distribution of gastric submucosal lesions. ∗ represents a statistically significant difference compared with the distribution in the stomach and cardia (*P* < 0.05).

**Figure 8:** Distribution of duodenal submucosal lesions.

**Figure 9:** Site and type of the upper gastrointestinal submucous lesions: (a) esophagus; (b) stomach; (c) duodenum.

**Figure 10:** Diagnostic results of ultrasound combined with gastroscope for the classification of upper gastrointestinal submucous lesions. ∗ shows a statistically significant difference compared with gastroscope examination (*P* < 0.05).

## Data Availability

The data used to support the findings of this study are available from the corresponding author upon request.
